The article "Optimization Research on Deep Learning and Temporal Segmentation Algorithm of Video Shot in Basketball Games" was retracted in 2023. Reasons: unreliable results or conclusions; concerns about the data; concerns about the results or conclusions; concerns about the peer review.

# Optimization Research on Deep Learning and Temporal Segmentation Algorithm of Video Shot in Basketball Games

**DOI:** 10.1155/2021/4674140

**Published:** 2021-09-06

**Authors:** Zhenggang Yan, Yue Yu, Mohammad Shabaz

**Affiliations:** ^1^Department of Physical Education, Zhongnan University of Economics and Law, Wuhan 430073, China; ^2^The Ministry of Public Basic Course, Wuhan Institute of Design and Sciences, Wuhan 430205, China; ^3^Arba Minch University, Arba Minch, Ethiopia; ^4^Chitkara University Institute of Engineering and Technology, Chitkara University, Rajpura, Punjab, India

## Abstract

The analysis of the video shot in basketball games and the edge detection of the video shot are the most active and rapid development topics in the field of multimedia research in the world. Video shots' temporal segmentation is based on video image frame extraction. It is the precondition for video application. Studying the temporal segmentation of basketball game video shots has great practical significance and application prospects. In view of the fact that the current algorithm has long segmentation time for the video shot of basketball games, the deep learning model and temporal segmentation algorithm based on the histogram for the video shot of the basketball game are proposed. The video data is converted from the RGB space to the HSV space by the boundary detection of the video shot of the basketball game using deep learning and processing of the image frames, in which the histogram statistics are used to reduce the dimension of the video image, and the three-color components in the video are combined into a one-dimensional feature vector to obtain the quantization level of the video. The one-dimensional vector is used as the variable to perform histogram statistics and analysis on the video shot and to calculate the continuous frame difference, the accumulated frame difference, the window frame difference, the adaptive window's mean, and the superaverage ratio of the basketball game video. The calculation results are combined with the set dynamic threshold to optimize the temporal segmentation of the video shot in the basketball game. It can be seen from the comparison results that the effectiveness of the proposed algorithm is verified by the test of the missed detection rate of the video shots. According to the test result of the split time, the optimization algorithm for temporal segmentation of the video shot in the basketball game is efficiently implemented.

## 1. Introduction

With the new development of computer technology, a video contains more abundant and vivid information and has become one of the important information carriers in the Internet [1]. The popularity of mobile terminals and the rise of video sites have made it easy to capture and share videos. The popularity of the video solves the need to process, analyze and deeply understand the massive amount of video data resources [2, 3]. There is various basketball events held every day in the world, and there are many videos recorded in the competition. Among them, the NBA is affecting the hearts of basketball fans all over the world [4]. The annual regular season and the playoffs not only attract the audience around the world, but even let the fans reach the level of sleepless nights. But normal work and life cannot satisfy watching every game [5], so the necessary screening needs to be done in order to select exciting clips for fans to enjoy. Manual screening satisfies the needs of fans to a certain extent, but the workload in this way will be large and people's preferences will be different [6, 7]. So, people are trying to study the mechanism to automatically extract the wonderful scenes of basketball games, to get rid of the dependence on labor, and try to provide personalized service for each fan [8]. All of this work must start with video segmentation. The quality of lens segmentation directly affects subsequent research. This is a crucial step. Focusing on the optimization of the temporal segmentation of the basketball video shot can pave the way for subsequent research and benefit more basketball video researchers [9].

In [10], the time domain segmentation algorithm based on the interframe difference distribution and gradual model is proposed. The threshold of the detected partial mutation frame is obtained by evaluating the interframe difference sequence of the video, and then, the entire interframe difference sequence is segmented. Repeat the same steps to get the abrupt frames of all video shots. In the aspect of detecting the gradation frame of the shots, according to the characteristics of the second-order difference of the gradation process and the gradation model, the correct gradation frame is obtained to optimize the segmentation of the video lens, but the missed detection rate of the algorithm is high. The temporal segmentation algorithm of the video shot in basketball games based on boundary classification is proposed in [11]. The view shots' boundary of the algorithm is the candidate boundary. Combined with the mute feature, the boundary is determined from both sound and video, and the final optimization result is obtained. However, the algorithm has a high missed detection rate so that the accuracy of lens segmentation optimization is low. In [12], the optimization of video shots' temporal segmentation algorithm based on the MapReduce model is proposed. A large number of data processing jobs are split into several independently executable map tasks for video decoding and feature extraction and to combine shot boundaries. The candidate shots' switching segments are filtered by adaptive thresholds for further detection, thereby optimizing the segmentation of the lens. However, the algorithm has longer split time and lower efficiency. The optimized segmentation algorithm based on new moving targets is proposed in [13] by introducing an adaptive kernel space. If the feature trajectories of the video belong to the same rigid object, they are mapped to the same point, and the embedded manifold denoising algorithm is used to segment the rigid and nonrigid video objects to obtain optimized results. The algorithm takes long time to split, and the efficiency of segmentation optimization is low.

The analysis of the video shot in basketball games and the edge detection of the video shot are the most active and rapid development topics in the field of multimedia research in the world. Video shots' temporal segmentation is based on video image frame extraction. It is the precondition for video application. Studying the temporal segmentation of basketball game video shots has great practical significance and application prospects.

The research box of the temporal segmentation optimization algorithm for the video shot of basketball games based on the histogram algorithm is as follows:

1. Analyze the concept and conversion type of the video shot of the basketball games. The conversion type of the shots can be divided into fade in, fade out, overlap, and sweep.
2. Using the threshold and the model method to detect the boundary of the video shot of the basketball games. The single-frame image of the video is processed, and the video image is reduced in dimension. The quantized dimensionality-reduced one-dimensional vector is used as a variable to perform histogram statistics and analysis on the video shots of basketball games, and the dynamic threshold is set to realize the temporal segmentation optimization of the video shots in basketball games.
3. The accuracy and efficiency of the optimized segmentation of the shots are tested to verify the effectiveness of the proposed method.
4. Summarize the research content.

The introduction to various methods and detailed literature has been presented in the current section. The various methods and techniques used for detection and interpretation of information from images and videos are presented in Section 2 under the heading “Materials and Methods.” Section 3 includes the work environment, and all the results obtained from experimentation are described in this section. Sections 4 and 5 represent the discussion and conclusion part of the study.

## 2. Materials and Methods

### 2.1. The Concept of Video Shots and Its Conversion Type

#### 2.1.1. Video Shot

The shot, as the most suitable unit of retrieval, is a sequence of frames that are continuously taken by the same camera. Most of the videos are connected because of the limited ability to describe the shot. These videos are mirrored to reflect what happens at different locations or times [14]. The typical structure used to organize the layers divides the video into 4 layers, as shown in Figure 1.

#### 2.1.2. The Division of Video Shots' Conversion Type

The conversion of the basketball video shot can be divided into two categories: shear and gradient. Switching into a shot directly converts to the next shot with no delay in time; the gradient includes stacking, fade in, fade out, and sweep. Among them, fade in and fade out can be used as the special case of stacking.

1. Fade in: gradually strengthen the picture
2. Fade out: slowly reduce the picture until it disappears
3. Overlay: while the previous lens is gradually weakened, the image of the next lens is gradually strengthened
4. Scanning: starting from a certain part of the screen, the previous lens is gradually replaced by the next lens

The above four types are the most commonly used and most studied basketball game video shot conversion types, and video editors often create some complex shots' conversion types based on subjective intentions.

### 2.2. Boundary Detection

#### 2.2.1. Threshold Method

The basic idea of the threshold method is that when the character *f*(*t*) of the basketball game video at a certain time *t* exceeds the threshold or is within a certain range, it is considered that the video shot changes at this time. One of the easiest ways to do this is to use the global threshold whose expression is as follows:

(1) $$\begin{array}{c} f\left(t\right)>T. \end{array}$$

In general, global thresholds that apply to all video and shot transitions do not exist. If the threshold is set too high, many missed conditions will occur, and setting the threshold too low will result in a higher false positive rate. Therefore, global thresholds [15] should be avoided as much as possible. An adaptive threshold approach is proposed to address the applicability of thresholds. The threshold of the moment *t* can be calculated by the following formula:

(2) $$\begin{array}{c} f\left(t\right)>T\left(t\right). \end{array}$$

The current dynamic threshold is calculated using the video feature values in the window consisting of the *w* frames before and after the current frame being examined. If the feature value of the checked frame is the maximum value within the window range and the ratio between the feature value and the average value of the feature values in the window is greater than the threshold *a*, then the frame is considered to have a shot shear, which uses the following expression:

(3) $$\begin{array}{c} f\left(t\right)=\max\left\{f\left(t+i\right)\right\},\;i\in \left[-w,w\right],\\ \frac{f\left(t\right)}{\max\left\{f\left(t+j\right)\right\}}>a,\;j\in \left[-w,w\right]\wedge j\neq 0. \end{array}$$

The adaptive threshold is expressed by probability, which minimizes the average error rate. The expression is as follows:

(4) $$\begin{array}{c} \frac{P\left(z|S\right)}{P\left(z|\bar{S}\right)}|{z=z}_{\left(k,k+l\right)}>\frac{1-P_{k}\left(S\right)}{P_{k}\left(S\right)}=\frac{1-P_{k}^{a}\left(S\right)P_{k}}{P_{k}^{a}\left(S\right)P_{k}}, \end{array}$$

where *S* and $\bar{S}$ are two hypotheses. Between the *k*th frame and the *k*+*l*th frame, the game video belongs to the same shot and the shot changes. *z*(*k*, *k*+*l*) is the nonsimilarity between the two frames. *P*(*z|S*) and $P\left(z|\bar{S}\right)$, respectively, indicate the probability of shot transition, and *P*_*k*_^*a*^(*S*) means the probability that *S* is true in the current situation.

At some point in time, the occurrence of shot shear shows the very prominent nonsimilarity feature, while the shot gradation occurs in a period of time, and the characteristics of each frame are not obvious. The double-threshold method is used to judge the shear and gradation of the shot. The expressions are

(5) $$\begin{array}{c} \text{Abrupt transition}:f\left(t\right)>T_{h},\\ \text{Gradual transition}:T_{l}<f\left(t\right)<T_{h}\wedge \sum f\left(t\right)>T_{h},t\in \left[t_{s},t_{e}\right]. \end{array}$$

Set two thresholds: the higher threshold *T*_*h*_ is used to detect the shear of the video shot in the basketball game. If the feature value of the video frame is greater than *T*_*h*_ at a certain time, it is considered that the shear occurs at this time; during the period from *t*_*s*_ to *t*_*e*_, if the feature values of all video frames are greater than the lower threshold *T*_*l*_ and the sum of their feature values is greater than *T*_*h*_, then it is considered that the video has a lens gradation during this time period.

#### 2.2.2. Model Method

In the process of fading out the black screen, the video is dimmed and darkened, and the color gradually becomes black. It can be described as

(6) $$\begin{array}{c} f_{\text{out}}\left(x,y,t\right)=g\left(x,y,t\right)a\left(t\right), \end{array}$$

where *f*_out_(*x*, *y*, *t*) means the color attribute of the *t* moment at the (*x*, *y*) position during the fade out process and *g*(*x*, *y*, *t*) represents the color attribute of the screen whose picture is faded out at the (*x*, *y*) position at the time *t*; when the faded picture is still, *g*(*x*, *y*, *t*) is the fixed value. *a*(*t*) represents a function that describes the color of the screen as the video shot fades out during the basketball game. During the process of fade out, *a*(*t*)=(1 − *t*)/*T*. The fade-in process of the shot is expressed by the following formula:

(7) $$\begin{array}{c} f_{m}\left(x,y,t\right)=g\left(x,y,t\right)\beta \left(t\right), \end{array}$$

where *β*(*t*)=*t*/*T*.

In the linear fade-in process, the video shot's stacking process can be seen as the combination of fade-out and fade-in processes:

(8) $$\begin{array}{c} f_{\text{dissolve}}\left(x,y,t\right)=f_{m}\left(x,y,z\right)+f_{\text{out}}\left(x,y,z\right). \end{array}$$

In order to detect the change model of the basketball game video footage, a constant graph is defined to describe the color change on each frame of the video shot:

(9) $$\begin{array}{c} \text{CI}\left(x,y,t\right)=\frac{f\left(x,y,t\right)}{f_{\text{dissolve}}\left(x,y,t\right)}, \end{array}$$

where CI(*x*, *y*, *t*)=−(1/*T*)*a*(*t*), which is a time function that is independent of the position (*x*, *y*). It can detect the gradual process of the video shot of the basketball game based on the constant graph curve. Both of the above methods can complete the detection of the video shot boundary of the basketball game.

### 2.3. Processing of Video Image Frames

The frame of the video image is further processed on the basis of the boundary detection. The processing of images of a single frame is roughly divided into the following steps:

One is to cut the source video image; the second is to extract the Canny boundary; the third is to optimize the boundary to remove impurities; the fourth is to search the curve in the optimized boundary and record the coordinate value of the point on the curve.

#### 2.3.1. Cutting

Through the above research, it can be found that the top of each frame of the image contains the viewer's picture. Influenced by factors such as clothes color or skin color, the Canny boundary is very messy, which seriously affects the subsequent research [16]. Therefore, before the further research begins, the source video image is cropped, which can reduce the amount of calculation and improve the accuracy of subsequent work.

The OTSU algorithm is used to binarize the extracted video frame image of the basketball game. The specific cropping scale is more suitable for retaining the bottom end of the source video image 7/10. The cut video of the basketball game video is shown in Figure 2.

#### 2.3.2. Canny Boundary

The Canny operator does not only determine whether a pixel is an edge point by the gradient operation. When determining whether a pixel is an edge point, it is necessary to consider the influence of other pixels at the same time. It is also not a simple boundary tracking. When looking for edge points, it needs to be judged based on the current and previously processed pixels [17]. It converts the edge detection problem into the maximum value of the detection function. The basic idea is to first smooth the image with a Gaussian filter and then use the finite difference of the first-order partial derivative to calculate the amplitude and direction of the gradient. The Canny boundary extracted from Figure 2 is shown in Figure 3.

#### 2.3.3. Optimization of Boundaries

The Canny edge indicator is an edge location administrator that utilizes a multistage calculation to distinguish a wide scope of edges in pictures. It was created by John F. Shrewd in 1986. Shrewd additionally created a computational hypothesis of the edge location clarifying why the strategy works. Canny edge detection is a strategy to extract helpful underlying data from images, and it drastically reduces the requirement of information and hence the processing. It has been broadly applied in different PC vision frameworks. Watchful has tracked down that the prerequisites for the utilization of edge recognition on assorted vision frameworks are somewhat comparable. In this way, edge recognition answer for addressing these necessities can be executed in a wide scope of circumstances.

The Canny boundary in Figure 3 contains target boundaries such as the three-point line and the forbidden line, but there are many interference boundary points at the same time, so it needs to be further optimized. The required boundaries are all in the form of two lines, and there is the relatively fixed distance between the two lines, which is no other point in the horizontal direction of the front and back [18]. Optimize the interference to the extracted Canny boundary and save the new data in a new result graph.

In Figure 3, the traversal from the first pixel to the end of the last pixel has the following steps:

1. Determine whether the pixel value of the current point is greater than zero. If it is greater than 0, proceed to step 2; otherwise, the left distance *d* is incremented by 1, and the corresponding point in the result graph is set to 0.
2. If the left distance *d* is greater than the distance threshold, proceed to step 3; otherwise, reset the left distance to 0, and set the corresponding point in the result graph to 0.
3. First set the left distance *d* to 0, and then, determine whether the number of nonzero points on the left boundary is less than 5. If yes, enter step 4; otherwise, set the value of the corresponding point in the result graph to the rightmost point of the left boundary to 0, and set the current point in Figure 3 to the next point of the rightmost point of the left boundary.
4. It is judged whether the number of zeros between the double lines is less than 6 and greater than 2. If yes, go to step 5. Otherwise, set the value of the rightmost point of the corresponding point to the zero-point sequence in the result graph to 0, and set the current point in Figure 3 to the next point of the rightmost point of the zero-point sequence.
5. Determine whether the number of nonzero points on the right boundary is less than 5. If it is less, the process proceeds to step 6. Otherwise, the value of the corresponding point in the result graph to the rightmost point of the right boundary is set to 0, and the current point in Figure 3 is set to the next point of the rightmost point of the right boundary.
6. Determine whether the number of subsequent zero points is greater than the distance threshold. If so, the value of the current point in Figure 3 is assigned to the current point in the result graph. Then, set the value of the next point of the current point to the rightmost point of the subsequent zero sequence to 0, and set the current point in Figure 3 to the next point of the rightmost point of the subsequent zero sequence. Finally, set the left distance to *d* for the number of subsequent zeros; otherwise, the value of the corresponding point in the result graph to the rightmost point of the subsequent zero sequence is set to 0, and the current point in Figure 3 is set to the next point of the rightmost point of the subsequent zero sequence. The result graph is the Canny boundary after optimization and decomplexation, which is recorded as *A*.

#### 2.3.4. Search Curve

The optimization boundary of the basketball game video shot is ideal, which has two characteristics:

1. The overall shape of the three-point line is similar to the parabola
2. The boundary points of the three-point line are relatively concentrated and relatively long, while most of the other boundary points are very scattered

Based on these two characteristics, the two methods are, respectively, designed to accurately locate the boundary curve that meets the requirements and record the coordinates of the points on the curve for later use [19].

*(1) Hough Transform*. The Hough transform is a component extraction method utilized in picture investigation, PC vision, and advanced picture processing. The reason for using this technique is that it helps to discover blemished cases of articles inside a specific class of shapes. This *d* technique is done in a boundary space, from which article up-and-comers are gotten as nearby maxima in a purported collector space that is expressly built by the calculation for processing the Hough change. Hough transform is used, and according to feature (1), the improved parabolic Hough transform is introduced which is capable of detecting the parabola contained in it, as shown in Figure 4.

The parabolic equation is

(10) $$\begin{array}{c} \left(x^{\prime }-x_{0}^{\prime }\right)=a^{\prime }\left(y^{\prime }-y_{0}^{\prime }\right),a^{\prime }\neq 0. \end{array}$$

After the derivative, it can be written as

(11) $$\begin{array}{c} \frac{d_{x^{\prime }}}{d_{y^{\prime }}}=2a^{\prime }\left(y^{\prime }-y_{0}^{\prime }\right). \end{array}$$

Take any point (*x*′, *y*′)on the parabola, and then, the tangential direction of the parabola at this point is *d*_*x*′_/*d*_*y*′_=2*a*′(*y*′ − *y*_0_′). Let the angle between the tangent of the parabola at this point and the *y*′ axis be *θ*; then, there is tan  *θ*=*d*_*x*′_/*d*_*y*′_. According to the above analysis, the following expression can be obtained:

(12) $$\begin{array}{c} \left\{\begin{array}{c} x_{0}^{\prime }=x{}^{\prime }-\frac{\tan^{2}\;\theta }{4a{}^{\prime }},\\ y_{0}^{\prime }=y{}^{\prime }-\tan\;\theta 2a{}^{\prime }. \end{array}\right) \end{array}$$

The improved parabolic Hough transform steps are as follows: set a three-dimensional accumulator array *A*(*a*′, *x*_0_′, *y*_0_′); for any edge point (*x*′, *y*′) in the basketball game video image, it is to use the edge gradient direction prediction value *θ* and change the value *a*′ to calculate (*x*_0_′, *y*_0_′) by formula (12), by voting for the accumulator array. After traversing all the edge points in this way, it is to look for the peak point of the accumulator to get the vertices and curvature of the parabola [20, 21].

*(2) Scanning Method*. According to proposed feature (2), the scanning method is adopted as follows:

  Initialize a basketball game video marker image and a new result image with the same size, and then, initialize a three-dimensional zero matrix, employed to record the coordinates of the point on the boundary curve. The first pixel point of A begins to traverse the entire video image.
  ② According to the value of the corresponding point in the basketball game video tag image to determine whether the current point in A is marked, if it is, then traverse the next point; otherwise, go to ③.
  ③ Determine whether the value of the current point is greater than 0. If yes, enter ④; otherwise, it will traverse the next point.
  ④ Determine whether there is a nonzero point in the area directly below the current point. If there is, increase the vertical length by 1, and set the current point to the nonzero point, continue to ⑤; otherwise, exit ④, and restore the current point to the original current point position. Go to ⑤ again.
  ⑤ Determine whether the longitudinal length from the current point is greater than the length threshold. If it is greater than the value, go to ⑥; otherwise, it will traverse the next point.

Determine whether there is a nonzero point in the area directly under the current point. If there is, assign the value of the current point to the corresponding point in the new result video image, and then, record the coordinate value of the point in the three-dimensional matrix (the first dimension represents the fixed boundary curve in the video image, the second dimension represents the fixed point on the current boundary curve, and the third dimension represents the coordinates of the current point), reset the corresponding point value in the marked video image to 1, and finally, set the current point to the nonzero point; go to ⑥; otherwise, exit ⑥ and restore the current point to the original current point position, and then, continue to traverse the next point.

Finally, the result map of the basketball game video is the boundary curve extracted from *A*, which can be used as the basis for subsequent video shot segmentation optimization.

### 2.4. Histogram Algorithm Based on the Optimization of Temporal Segmentation Algorithm for Video Shot of Basketball Games

Based on the above analysis, the overall framework for video segmentation of basketball games is established. The video data is converted from the RGB space to the HSV space by the boundary detection of the video shot of the basketball game and the processing of the image frames, in which the histogram statistics are used to reduce the dimension of the video image, and the three-colors components in the video are combined into a one-dimensional feature vector to obtain the quantization level of the video. The one-dimensional vector is used as the variable to perform histogram statistics and analysis on the video shot and to calculate the continuous frame difference, the accumulated frame difference, the window frame difference, the adaptive window's mean, and the superaverage ratio of the basketball game video. The calculation results are combined with the set dynamic threshold to optimize the temporal segmentation of the video shot in the basketball game.

The overall framework of the temporal segmentation of the basketball game video shot is shown in Figure 5.

The basketball game video is generally represented by RGB values, which need to be converted from RGB space to HSV space. When performing histogram statistics, the amount of calculation is too large, so it needs to be dimension-reduced. According to the human visual resolution, the color *H* is divided into 8 parts, and the saturation *S* and the brightness *V* space are, respectively, divided into 3 parts, and the following expression is obtained:

(13) $$\begin{array}{c} H=\left\{\begin{array}{c} 0\text{ if }h\in \left[316,20\right],\\ 1\text{ if }h\in \left[21,40\right],\\ 2\text{ if }h\in \left[41,75\right],\\ 3\text{ if }h\in \left[76,155\right],\\ 4\text{ if }h\in \left[156,190\right],\\ 5\text{ if }h\in \left[191,270\right],\\ 6\text{ if }h\in \left[271,295\right],\\ 7\text{ if }h\in \left[296,315\right], \end{array}\right)\\ S=\left\{\begin{array}{c} 0\text{ if }s\in \left[0,0.2\right],\\ 1\text{ if }s\in \left[0.2,0.7\right],\\ 2\text{ if }s\in \left[0.7,1\right], \end{array}\right)\\ V=\left\{\begin{array}{c} 0\text{ if }v\in \left[0,0.2\right],\\ 1\text{ if }v\in \left[0.2,0.7\right],\\ 2\text{ if }v\in \left[0.7,1\right]. \end{array}\right) \end{array}$$

According to the above quantization level, the three-color components in the basketball game video are combined into one-dimensional feature vector, and the expression is as follows:

(14) $$\begin{array}{c} G=HQ_{S}Q_{V}+SQ_{V}+V, \end{array}$$

where *Q*_*S*_and *Q*_*V*_ represent the quantization levels of the components *S* and *V*, respectively, and *Q*_*S*_=3, and *Q*_*V*_=3. It can be converted to

(15) $$\begin{array}{c} G=9H+3S+V, \end{array}$$

While the three components of *H*, *S*, and *V* are distributed on the one-dimensional vector *G*, the value of *G* ranges from [0,1,…, 71]. Using the one-dimensional vector *G* after the quantized dimensionality reduction as a variable, the histogram statistical analysis of the basketball game video shot also needs to calculate the continuous frame difference of the basketball game video, the accumulated frame difference, the window frame difference, the adaptive window's mean, and superaverage ratio.

#### 2.4.1. The Continuous Frame Differences

Provided {*I*_1_, *I*_2_, *I*_3_,…, *I*_*n*_} as a sequence of video frames for the basketball game video, the corresponding histograms are {*h*_1_, *h*_2_, *h*_3_,…, *h*_*n*_}. The continuous frame difference of the basketball game video is calculated as the difference value of the histograms of consecutive adjacent frames. The calculation formula is

(16) $$\begin{array}{c} HD_{i\prime }\left(G\right)=\sum_{G=0}^{71}\left|h_{i\prime }\left(G\right)-h_{i\prime -1}\left(G\right)\right|. \end{array}$$

In the formula, *HD*_*i*′_(*G*) represents the histogram difference between the video frame *i*′ − 1 and the frame *i*′ of the basketball game, which is called the continuous frame difference of the frame *i*′.

#### 2.4.2. The Accumulated Frame Differences

The accumulated frame difference of the basketball game video refers to the *i*′th frame of image *I*_*i*′_ in the video sequence as the reference frame, and the histogram difference value between each frame and the reference frame is calculated. So, the obtained difference value of the series is the accumulated frame difference of the *i*′th frame *I*_*i*′_ image in the basketball game video as follows:

(17) $$\begin{array}{c} {\text{HDA}}_{i^{\prime }j^{\prime }}\left(G\right)=\sum_{G=0}^{71}\left|h_{j\prime }\left(G\right)-h_{i^{\prime }}\left(G\right)\right|, \end{array}$$

where HDA_*i*′*j*′_(*G*) represents the histogram difference value of the basketball game video between frame *I*_*j*′_ and frame *I*_*i*′_, *j*′=*i*′+*k*′(*k*′=1,2,3,…).

#### 2.4.3. Window Frame Difference

It refers to the ratio of the continuous frame difference of each frame to the continuous frame difference of the first window frame in a window, and the maximum value of the ratio is the frame difference of the window. Its expression is

(18) $$\begin{array}{c} FW_{n}=\max\left\{\frac{HD_{j^{\prime }}\left(G\right)}{HD_{i^{\prime }}\left(G\right)}\right\}, \end{array}$$

where *FW*_*n*_ is the window frame difference for the video, *n* is the size of window, *I*_*i*′_ is the start frame of the window, and *I*_*j*′_ is the sequence of frames within the window, *j*′=*i*′+*k*′(*k*′=1,2,…, *n* − 1).

#### 2.4.4. Mean Value of the Adaptive Window

It refers to adaptively opening a window of *n* frame size at the assumed gradient start frame position, taking the mean value of each successive frame difference in the window. Its calculation formula is as follows:

(19) $$\begin{array}{c} WA_{n}=\frac{\sum_{j^{\prime }=0}^{n-1}HD_{j^{\prime }}\left(G\right)}{n}, \end{array}$$

where *WA*_*n*_ is the mean value of the adaptive window of the window with *n* frame.

#### 2.4.5. Supermean Ratio

It means that, in the set window, the continuous frame difference of each frame image is larger than the average of the adaptive window mean. The ratio obtained compared with the window size is the superaverage ratio of the window. The calculation formula is

(20) $$\begin{array}{c} \eta_{n}=\frac{\sum_{j\prime =0}^{n-1}\partial_{j^{\prime }}}{n},\\ \partial_{j^{\prime }}=\left\{\begin{array}{cc} 1, & \text{if }HD_{j^{\prime }}\left(G\right)>WA_{n},\\ 0, & \text{if }HD_{j^{\prime }}\left(G\right)\leq WA_{n}, \end{array}\right) \end{array}$$

where *η*_*n*_ represents the window's superaverage ratio and ∂_*j*′_ represents the ratio factor. Through the calculation of the continuous frame difference, the accumulated frame difference, the window frame difference, the adaptive window's mean, and the superaverage ratio of the basketball game video, the time segmentation of the video footage of the basketball game is paved, and the video shot of the basketball game is analyzed, in order to do segmentation optimization.

The change of the shots refers to the switching between one shot and the other shot. Through the calculation of equation (16), the continuous frame difference *HD*_*i*′_(*G*) of the basketball game video sequence can be obtained in turn, and two dynamic thresholds *T*_1_′ and *T*_2_′ are set, where *T*_1_′=*b∗HD*_*i*′−1_ and *T*_2_′=*b∗HD*_*i*′+1_, *b* are coefficients. Combining the dynamic threshold with the above calculation results can optimize the time domain segmentation of the video shot of the basketball game. The expression is

(21) $$\begin{array}{c} L=\left(\eta_{n}+WA_{n}+FW_{n}+H\;DA_{i^{\prime }j^{\prime }}\left(G\right)+HD_{i^{\prime }}\left(G\right)\right)\cdot T_{1}^{\prime }T_{2}^{\prime }+\delta . \end{array}$$

The optimal solution *δ* is obtained, and the optimization of the temporal segmentation of the video shot in the basketball game is completed.

## 3. Results

The experiment selects the CPU with 2 GB memory, the running software is MATLAB, and the running system is Windows7. In order to verify the effectiveness of the proposed algorithm, a temporal segmentation optimization algorithm based on the histogram algorithm, a temporal segmentation optimization algorithm based on interframe difference distribution and gradual model, and a temporal segmentation optimization algorithm based on boundary categorization are used to test the missed detection rate (ignoring the effect of the ratio factor and setting the ratio factor to be constant expressed in *μ*), and the result is shown in Figure 6.

Analysis of Figure 6(a) shows that the missed detection rate of the video shot corresponding to the video shot number 1 to 6 of the basketball game is between 0 and 40%, and the fluctuation is not large. It can be seen from Figure 6(b) that the video detection rate of the video shot corresponding to the video shot number 1 to number 6 of the basketball game is relatively high, ranging from 60% to 100%, and the highest missed detection rate is close to 100%. In Figure 6(c), the highest rate of missed detection of the basketball video shot is close to 80%. Based on the data presented in Figures 6(a)–6(c), it is clearly seen that the missed detection rate third method is low. Thus, it may be stated the detection rate of the basketball game video shot of the proposed algorithm is low, which indicates that the algorithm has higher accuracy in optimizing the temporal segmentation of the basketball game video shot.

Using the segmentation time of the video shot to further study the efficiency of video shot temporal segmentation optimization, the shorter the segmentation time is, the higher the efficiency is, and the test results are shown in Figure 7.

In Figure 7, method 1 represents the algorithm proposed in this paper, method 4 represents the optimization segmentation algorithm based on MapReduce, and method 5 represents optimization segmentation algorithm based on the new moving object. As can be seen from Figure 7(a), the shot split time of 12 iterations is less than 0.6 s. In Figures 7(b) and 7(c), the shot split time of 12 iterations is between 0.5–0.9 s and 0.5–1.0 s, respectively. The longest split time of Figure 7(c) is close to 1 s. The comparison results show that the proposed algorithm has the shortest time to segment the video shot of the basketball game, which indicates that the algorithm is more efficient in optimizing the temporal segmentation of the basketball game video shot.

## 4. Discussion

Through the test of the missed detection rate of the basketball game video shot, the accuracy of the video shot temporal segmentation optimization of the proposed algorithm is verified. Figure 6 represents the missed detection rate (in percentage) for the three methods, the proposed and other two methods. The results indicate that the proposed method has lesser missed detection time than the other method. Also, Figure 7 indicates that the split time of the proposed method is shortest. On this basis, the time used for shot segmentation is further compared. The above two experiments not only verify the accuracy of the temporal segmentation optimization of the basketball game video shot of the proposed algorithm but also efficiently complete the temporal segmentation optimization of the basketball game video shot.

## 5. Conclusions

Based on the histogram algorithm, the research focuses on the optimization of the temporal segmentation algorithm for video shot of basketball games. It is divided into two stages: using the missed detection rate of the basketball game video shot to test the accuracy of temporal segmentation optimization, which verifies that the proposed algorithm can accurately optimize the video segmentation. Using the segmentation time of the video shot of the basketball game to test the efficiency of temporal segmentation optimization, and it is verified that the proposed algorithm can efficiently complete the temporal segmentation optimization of the basketball game video shot.

## Figures and Tables

**Figure 1:** The structure of the basketball game video data.

**Figure 2:** Cut video shot.

**Figure 3:** Extracted Canny boundary.

**Figure 4:** Hough transform of improved parabola.

**Figure 5:** The overall frame of the video shot temporal segmentation.

**Figure 6:** Video shot missed detection rate. (a) Method 1's missed detection rate. (b) Method 2's missed detection rate. (c) Method 3's missed detection rate

**Figure 7:** Split time of the video shot. (a) Split time of method one. (b) Split time of method four. (c) Split time of method five.

## Data Availability

The data used to support the findings of the study are available from the corresponding author upon request.
